RETRACTED

# Use of Platelet-Rich Fibrin in the Treatment of Periodontal Intrabony Defects: A Systematic Review and Meta-Analysis

**DOI:** 10.1155/2021/6669168

**Published:** 2021-02-04

**Authors:** Liang Chen, Yi Ding, Guoping Cheng, Shu Meng

**Affiliations:** ^1^National Clinical Research Center for Oral Diseases, West China Hospital of Stomatology, Sichuan University, Chengdu, Sichuan 610041, China; ^2^State Key Laboratory of Oral Diseases, Sichuan University, Chengdu, Sichuan 610041, China; ^3^Department of Periodontology, West China College of Stomatology, Sichuan University, Chengdu, Sichuan 610041, China

## Abstract

**Background:**

Platelet-rich fibrin (PRF) is a kind of autologous platelet concentrate which is easy to obtain and cheap. In recent years, it has been studied to improve the effect of periodontal regeneration. However, few studies have systematically evaluated the complementary effect of PRF in the treatment of intrabony defects. The present review is aimed at systematically assessing the effects of PRF on clinical and radiological outcomes of the surgical treatment of periodontal intrabony defects.

**Methods:**

The protocol was registered at PROSPERO (International Prospective Register of Systematic Reviews) as CRD42020206056. An electronic search was conducted in MEDLINE, Cochrane, and EMBASE databases. Only randomized clinical trials were selected. Systematically healthy patients with two or three walls of intrabony defects were considered. Intrabony defect (IBD) depth reduction and bone fill (BF) % were set as primary outcomes while probing depth (PD) reduction, clinical attachment level (CAL) gain, and gingival margin level (GML) gain were considered as the secondary outcome. When possible, a meta-analysis was performed.

**Results:**

Eighteen articles fulfilled the inclusion criteria, and seventeen studies were quantitatively analyzed. Of 17 studies, four were rated as high risk of bias and thirteen as the moderate risk of bias. Two comparisons were set: (1) open flap debridement (OFD) combined with PRF and OFD alone and (2) bone grafting (BG) combined with PRF and BG alone. Compared to OFD alone, OFD+PRF showed significantly greater in all primary and secondary outcomes. Compared to BG alone, BG+PRF showed significantly greater in IBD depth reduction, PD reduction, CAL gain, and GML gain.

**Conclusions:**

The use of PRF was significantly effective in the treatment of periodontal intrabony defects. The benefit of OFD+PRF may be greater than BG+PRF. PRF can promote early wound healing in periodontal surgery. As all included studies were not at low risk of bias, well-designed RCTs having a high methodological quality are needed to clarify the additional effectiveness of PRF in the treatment of intrabony defects in the future.

RETRACTED

## 1. Introduction

Periodontitis is defined as a chronic inflammatory disease caused by periodontopathic bacteria and is characterized by inflammation and the progressive destruction of tooth-supporting tissues [1], which is the major cause of tooth loss in adults. Regeneration of the periodontal tissues and a return to clinically healthy status are the ultimate goals of the treatment of periodontal diseases. Periodontal regeneration involves the reconstruction of alveolar bone, periodontal ligament, and cementum [2], which is a multifactorial and complex process. Alveolar bone resorption is a typically pathological manifestation of periodontal diseases and a signature event in the diagnosis, which can cause vertical and/or horizontal bone defects and contribute to tooth mobility and even the loss of tooth. Horizontal bone defects are usually difficult to regenerate, while vertical bone defects, especially intrabony defects, are considered to have good regeneration potential. A variety of different surgical techniques, usually including guided tissue regeneration, various types of bone grafts or bone substitutes techniques, growth and differentiation factors, root surface demineralization, enamel matrix proteins or various combinations thereof, have been investigated to regenerate periodontal tissues [3, 4].

Platelet *α*-granules contain a great number of growth factors: vascular endothelial growth factor (VEGF), epidermal growth factor (EGF), platelet-derived growth factor (PDGF), transforming growth factor (TGF), platelet factor interleukin (IL), platelet-derived angiogenesis factor (PDAF), insulin-like growth factor (IGF), and fibronectin [5–7], which play an important role in wound healing and regeneration. In recent years, autologous platelet concentrate has been widely used in oral tissue regeneration [8] and wound healing [9]. Platelet-rich plasma (PRP) is the first generation of platelet concentrate, mainly produced by two-step centrifugation and the addition of bovine thrombin and calcium to activate platelets and release growth factors [10]. However, growth factors in PRP are released quickly. Platelet-rich fibrin (PRF) was developed in France by Choukroun et al. [11], and second-generation platelet concentrate is prepared by using a simplified regimen compared to PRP, no biochemical handling of blood or use of any gelling agent like calcium chloride and no risks associated with the use of bovine thrombin [12, 13]. Besides, PRF has a three-dimensional fibrin architecture [14], forming a scaffold to maintain growth factors, in which growth factors are released for more than 7 days [15].

RETRACTED

The use of PRF in periodontal regeneration procedures may have potential benefits. A systematic review and meta-analysis [16] reported the effect of autologous platelet concentrate on the treatment of intrabony defects (IBD), but PRF was not evaluated. Castro et al. [17] reported a meta-analysis of 6 studies until 2016, but only three parameters including PD reduction, CAL gain, and bone fill were evaluated, and the evaluation is not detailed enough concerning intrabony defects. After that, more RCTs have been published, so it is necessary to evaluate the effect of PRF in the treatment of periodontal intrabony defects with detailed hard and soft tissue parameters.

The present systematic review and meta-analysis is primarily aimed at evaluating whether PRF could provide additional benefits for intrabony defect, by comparing the clinical and radiological parameters between periodontal surgery alone and periodontal surgery with using PRF in the treatment of intrabony defects.

## 2. Materials and Methods

### 2.1. Protocol and Registration

This study was conducted based on the guidelines of the Cochrane Handbook for Systematic Reviews of Interventions [18] and is reported following the Preferred Reporting Project Guidelines for Systematic Review and Meta-analysis (PRISMA) statement [19]. The protocol of this systematic review and meta-analysis was registered on the PROSPERO (CRD42020206056).

### 2.2. Eligibility Criteria

The inclusion criteria were set according to PICOS question: the participants (P) included systemically healthy adults who have suffered periodontal diseases with periodontal intrabony defects; the intervention (I) was periodontal surgery with the use of PRF; the comparison (C) was periodontal surgery without the use of PRF; the outcomes (O) contained radiographic parameters including IBD depth reduction and vertical bone fill (BF) % and clinical parameters including probing depth (PD), clinical attachment level (CAL), and gingival margin level (GML); the study (S) was only considered to be randomized controlled trials (RCTs) with blindness.

The exclusion criteria were as follows: (1) patients with systematic diseases or pregnancy or lactation for women; (2) smoker or using drugs known to affect the outcomes of periodontal therapy; (3) absent or uncompleted periodontal initial therapy before periodontal surgery; (4) one-wall defects included; (5) studies investigating any other oral surgical intervention like tooth extraction, implant therapy, treatment of jawbone defects, odontogenic cysts, and periapical surgery.

### 2.3. Information Sources and Search Strategy

Three electronic databases were searched without limits regarding publication date or status: MEDLINE via PubMed, EMBASE, and Cochrane Central Register of Controlled Trials (CENTRAL). Only articles published in English were eligible. The last search was conducted on 16 November 2020. The search strategy was performed by combining (Mesh Terms OR Key Words) and using the following terms: “platelet concentrates” OR “platelet-rich fibrin” OR “PRF.” In addition, OpenGrey (http://www.opengrey.eu) and Grey Literature Report (http://www.greylit.org) were used to supplement the search for grey literature by using the term “platelet-rich fibrin.”

RETRACTED

### 2.4. Study Selection and Data Collection Process

The titles and abstracts obtained from the first search were screened independently by the two reviewers (Liang Chen and Guoping Cheng). After the initial assessment, all full texts of the eligible articles were obtained and examined by both reviewers. Any disagreement in the final selection was resolved by open discussion between the two reviewers and by consulting a third author (Shu Meng).

Data from the studies included in the final selection were extracted independently by the two reviewers (Liang Chen and Guoping Cheng) and finally cross-checked. The extracted data information was as follows: (1) general characteristics: author, publication year, study design, duration, groups, country, and setting (university setting or private practice setting); (2) patient characteristics: number of patients and sites, sex, mean age of the patients, and smoking; (3) intrabony defect features: number of sites in each group, type of arch (maxilla, mandible, or both), tooth type, and walls of IBDs; (4) outcomes: probing depth (PD) reduction, clinical attachment level (CAL) gain, gingival margin level (GML) gain, IBD depth (alveolar bone crest to base of the defect) reduction, and vertical bone fill (BF) %.

### 2.5. Risk of Bias in Individual Studies and across Studies

The risk of bias was assessed by both reviewers (Liang Chen and Guoping Cheng) according to the Cochrane Handbook for Systematic Reviews of Interventions [18]. Seven quality criteria were verified: (1) random sequence generation (selection bias), (2) allocation concealment (selection bias), (3) blinding of participants and personnel (performance bias), (4) blinding of outcome assessment (detection bias), (5) incomplete outcome data (attrition bias), (6) selective outcome reporting (reporting bias), and (7) other bias.

After the quality assessment, individual studies were categorized as being at low, high, or moderate risk of bias according to the following criteria: (1) low risk of bias: all domains were at low risk of bias; (2) high risk of bias: one or more domains were at high risk of bias; (3) moderate risk of bias: one or more domains were at unclear risk of bias and no high risk of bias. Heterogeneity across studies was characterized using Cochran-*Q* statistic and *I*^2^ statistic tests.

RETRACTED

### 2.6. Data Analysis

Data from the included studies were pooled to estimate the effect size, expressed as mean difference (MD) and 95% confidence interval (CI). When the homogeneity between the studies was good (*P* ≥ 0.10 and *I*^2^ ≤ 50%), the fixed-effects model was used for data merging. On the contrary, when *P* < 0.10 and *I*^2^ > 50%, the random-effects models were used. Data analyses were performed using the RevMan software [20].

## 3. Results

### 3.1. Study Selection

A total of 391 related articles (78 in PubMed, 227 in EMBASE, and 86 in Cochrane Central Register of Controlled Trials) were obtained, and none result was found in OpenGrey and Grey Literature Report. Then, 112 duplicate literatures were excluded, and 29 articles of the remaining 278 articles were screened by reading the titles and abstracts. After reading carefully the full text, 18 RCTs fulfilled the inclusion criteria and were selected for qualitative analysis, and 17 of them were included for meta-analysis as mean changes data could not be extracted from one study. A PRISMA flow diagram that depicts this selection process is displayed in Figure 1.

### 3.2. Study Characteristics

The general characteristics of the 18 studies included are displayed in Table 1. All the 18 studies were RCTs, of which 9 [13, 21–28] were split-mouth design and 9 [29–37] were parallel arm design. All the subjects were systematically healthy adults who suffered periodontitis with intrabony defects, except for one study [37] in which participants had periodontal-endodontic lesions with intrabony defects. And the type of intrabony defects is two-wall or three-wall. Further, all studies did not recruit smokers. In each study, periodontal initial therapy was performed before periodontal surgery. No study performed a minimally invasive surgery, and open flap debridement was used in all studies. The use of PRF as sole biomaterial or in combination with bone substitute grafting was used in the test group, while OFD alone or combined with bone substitute grafting was used in the control group. In terms of results assessment, there was no measurement calibration reported in two studies [13, 37]. Customized acrylic stents with grooves were used for measurement of clinical parameters using a periodontal probe, except for the two studies [13, 23] using a periodontal probe only. Intraoral standardized radiographs using the paralleling technique were used for radiological measurements except one study [24] using CBCT. Participants maintained proper oral hygiene during the follow-up period of 6-12 months in all studies. Additionally, all included studies were conducted in a university setting from India, Egypt, or Turkey.

RETRACTED

### 3.3. Risk of Bias in Individual Studies

The risk of bias within selected studies is shown in Figure 2. All studies reported randomization of sequence generation with coin tossing or computer-generated tables. Concerning allocation concealment, all studies did not use methods such as opaque envelopes. However, one study [25] indicated clearly that it was randomized immediately before surgical operation, so neither the participants nor the researchers could predict the allocation results. It can be considered that the allocation concealment is sufficient allocation hiding in this study, and there is no adequate allocation hiding in the others except for this study. In terms of blinding, as it is a surgical operation, the personnel cannot be blind. All the included studies blinded the outcome assessment, one [25] of which did not blind the participants, and six studies [13, 22, 24, 27, 28, 36] did not state whether the participants were sufficiently blind. Incomplete outcome data were reported in three studies [25, 31, 35] with either imbalance in numbers or reasons for missing data across intervention groups. No selective reporting was found. Other bias was found in the studies of Rosamma et al. [13] and Ustaoğlu et al. [37] for no measurement calibration. According to the Cochrane Collaboration's tool for assessing the risk of bias, thirteen [21–24, 26–30, 32–34, 36] of the selected studies presented a moderate risk of bias, whereas five studies [13, 25, 31, 35, 37] exhibited a high risk of bias.

### 3.4. Synthesis of Results

Among the included 18 studies, 14 compared the effects of PRF with that of OFD alone. In terms of soft tissue parameter, one study [22] showed that there was no statistically significant difference in PD reduction between the control group and the experimental group, and no significant difference in CAL improvement among the three studies. Except that, remaining 13 studies showed that the use of PRF significantly improved CAL and reduced PD compared with the control group. Additionally, only 10 of the 14 studies reported the GML changes, and all studies showed that the GML changes of the PRF group were better than that of the control group except for one study [22]. In terms of hard tissue parameter, IBD depth reduction, and BF%, 12 studies [13, 22, 23, 29–37] that have reported the two data showed that the effect of the use of PRF was better than OFD only.

RETRACTED

Four of the 18 studies compared the effects of BG combined with PRF and bone grafting without PRF. Agarwal et al. [21] reported when 12 months after operation, the BG combined with PRF group exhibited statistically significantly greater changes compared with the BG group in PD reduction, CAL gain, GML gain, IBD depth reduction, and bone fill%. Bodhare et al. [24] reported when 6 months after operation, BG combined with PRF is found to be significantly greater in the gain in CAL and IBD depth reduction and more effective in PD reduction although not significant, as compared to treatment with BG alone in periodontal intrabony defects. No significant clinical differences between BG group and BG combined with PRF group during six months or nine months were reported in the research by Gamal et al. [25]. In the six-month study of Sezgin et al. [27], gain in CAL was significantly greater in the test group than in the control group, whereas no intergroup differences were observed in PD reduction, GML changes, and IBD depth reduction.

Moreover, two articles have assessed the effect of PRF for wound healing. In the research of Patel et al. [26], at 7 days after surgery, all 13 sites in the test group (OFD+PRF) showed perfect healing (i.e., score 1 of wound healing index [100%]), and in the control group, only five sites showed perfect healing (i.e., score 1 of wound healing index [38%]). The difference between test and control groups at 7 days was significant (*P* = 0.003). At the end of 14 days, all sites in the test group and nine sites in the control group showed perfect healing with a score 1 of WHI (70%) with no statically significant difference (*P* = 0.21). In the study of Rosamma et al. [13], after 7 days, visual analog scale was used to assess the patient experience and the initial soft tissue healing with the two treatment modalities. The result showed that, compared to OFD alone, the use of PRF significantly reduced the postoperative pain and discomfort after periodontal surgery and significantly accelerated periodontal wound healing.

As mean change data could not be extracted from the study of Gamal et al. [25], a total of 17 RCTs were quantitatively analyzed. The primary outcomes were IBD depth reduction and bone fill%, and the secondary outcomes were the changes in PD, CAL, and GML. PRF as the only implant substances or combined with bone graft substitute, other bone stimulating substances such as ALN, ATV, MF, and RSV were not included in this analysis. In this meta-analysis, two comparisons are set up as follows.

#### 3.4.1. OFD+PRF vs. OFD Alone

In the primary outcomes (Figure 3), the heterogeneity was high in IBD depth reduction (*I*^2^ = 93%) and BF% (*I*^2^ = 92%), so a random-effects model was used. A statistically significantly greater in IBD depth reduction (mean difference: 1.81 mm; 95% CI: 1.53 to 2.08) with additional PRF in OFD was found. Similarly, a statistically significant beneficial effect of BF% (mean difference: 39.56%; 95% CI: 36.73 to 42.38) was found in the OFD+PRF group.

RETRACTED

In the secondary outcomes (Figure 4), the meta-analysis showed that the clinical parameters of OFD+PRF group were better than those of OFD alone group. There are statistically significant differences in PD reduction (mean difference: 1.18 mm; 95% CI: 0.94 to 1.42), CAL gain (mean difference: 1.25 mm; 95% CI: 0.93 to 1.57), and GML gain (mean difference: 0.42 mm; 95% CI: 0.32 to 0.53), with high heterogeneity across the studies (*I*^2^ = 87%, 90% and 92%, respectively).

#### 3.4.2. B +PRF vs. BG Alone

There were only three studies [21, 24, 27] in this comparison (Figure 5). No evidence of heterogeneity was found (*I*^2^ = 0.0%) across the studies in IBD depth reduction, PD reduction, and CAL gain, so a fixed-effects model was applied. Random-effects model was used in GML gain with a high heterogeneity (*I*^2^ = 52%). Only one article reported BF% data, so meta-analysis was only conducted in IBD depth of primary outcomes. The results show that a greater IBD depth reduction for the BG+PRF group was found than BG alone group, and the difference was statistically significant (mean difference: 0.92 mm; 95% CI: 0.66 to 1.18).

As for the secondary outcomes, compared with the BG alone group, the BG+PRF group showed more statistically significant advantages in PD reduction (mean difference: 0.52 mm,;95% CI: 0.21 to 0.82), CAL gain (mean difference: 1.09 mm; 95% CI: 0.77 to 1.41), and GML gain (mean difference: 0.69 mm; 95% CI: 0.31 to 1.06).

### 3.5. Risk of Bias across Studies

The publication bias was evaluated by the visual symmetry of the funnel plot (Figure 6). The studies with large sample size and high accuracy were distributed at the top of the funnel plot and concentrated in the vertical line, while other studies were evenly distributed on both sides. The shape of funnel plot was approximately symmetrical, indicating no obvious publication bias.

## 4. Discussion

### 4.1. Summary of Evidence

This systematic review and meta-analysis focused on evaluating the effectiveness of surgical treatment of periodontal bone defects with PRF, including clinical and radiological parameters. Clinical scenarios involving implants were beyond the scope of this review. The results of this meta-analysis revealed that OFD combined with PRF is more effective than OFD procedures alone, radiographically in IBD depth reduction by 1.81 mm (95%CI = 1.53, 2.08) and vertical bone fill% by 39.56% (95%CI = 36.73, 42.38), as well as clinically in PD reduction by 0.52 mm (95%CI = 0.21, 0.82), CAL gain by 1.25 mm (95%CI = 0.93, 1.57), and GML gain by 0.42 mm (95%CI = 0.32, 0.53). In addition, BG combined with PRF found to be more effective than BG procedure alone radiographically in IBD depth reduction by 0.92 mm (95%CI = 0.66, 1.18), as well as clinically in PD reduction by 0.52 mm (95%CI = 0.21, 0.82), CAL gain by 1.09 mm (95%CI = 0.77, 1.41), and GML gain by 0.69 mm (95%CI = 0.31, 1.06). Furthermore, the qualitative analysis showed that, after 7 days, better wound healing occurred with the use of PRF.

RETRACTED

Only one meta-analysis has been reported to evaluate the additional effect of PRF in the treatment of intrabony defects before. The meta-analysis of Castro et al. [17] only compared OFD+PRF to OFD alone, including a total of 6 studies until 2016. Comparing to OFD alone, OFD+PRF showed greater improvement in IBD depth reduction by 1.65 mm (95%CI = 0.99, 2.31), PD reduction by 1.1 mm (95%CI : 0.62, 1.58), and CAL gain by 1.24 mm (95%CI : 0.59, 1.89). It was indicated that OFD+PRF is more effective than OFD alone, which is in accordance with our results. A meta-analysis [38] showed that OFD+1% alendronate+PRF was even better than OFD+PRF. However, GML and BF% changes were not assessed in the study of Castro et al. Interestingly, our study revealed that PRF has certain benefits for GML gain in both OFD and BG surgery. Besides, we found that the combination of bone grafting with PRF will further generate statistically better changes of soft and hard tissue than BG alone.

The use of PRF is also beneficial to other oral tissue regeneration. Based on recent systematic reviews and meta-analysis, OFD+PRF demonstrated better results than OFD alone in grade II furcation treatment [39]. In terms of gingival recession, Moraschini and Barboza Edos [40] have reported in 2016 that the use of PRF membranes did not improve the root coverage, keratinized mucosa width, or CAL of Miller classes I and II gingival recessions compared with the other treatment modalities. On the contrary, the meta-analysis of Li et al. [41] and Panda et al. [42] suggested that PRF when used in addition to coronally advanced flap (CAF) showed favorable results for the treatment of gingival recession defects. Moreover, He et al. [43] reported that local application of PRF after lower third molar extraction was a valid method for relieving pain and 3-day postoperative swelling and reducing the incidence of alveolar osteitis.

### 4.2. Limitations

In order to adhere to high methodological standards and to maximize the clinical applicability of the results reported in this review, stringent inclusion criteria were adopted. In terms of study design, split-mouth design and parallel design were included in this review, because recent evidence showed that both of them are equally effective [44]. In regard of participants, studies including smokers are excluded, because smoking is a clear risk factor of periodontal diseases [45] and significantly affects the outcome of periodontal regeneration surgery [4, 46]. The type of intrabony defects was limited in only two or three walls, because the number of remaining bony walls was found to be correlated positively with regeneration potential in grafting procedures [47], and one-wall defect is a risk factor for failure (odds ratio [OR] ≥ 10.4) [48]. In the blind method, we require that outcome assessments must be blinded. On the one hand, due to surgery procedures, operation physicians could not be blinded; on the other hand, the final measurement is done manually regardless of clinical or radiographical measurement, and the results will be greatly affected by the accessors. Thus, blinding for the outcome assessment was of great importance, and studies without blind method were excluded. Although screening programs were stringent, there was still no risk of low bias in this review, and at least one ambiguous bias risk emerged in all studies, mainly in the domain of allocation concealment and blinding of participants.

RETRACTED

In the quantitative analysis of the effect of PRF on periodontal surgery, the heterogeneity among the studies was as high as the meta-analysis of Castro et al. [17], Tarallo et al. [39], Panda et al. [42], Li et al. [38], and Li et al. [41]. Heterogeneity may come from different clinical research methodology and implementation processes. (1) Different preparation and usage methods of PRF: the preparation of PRF entirely depends on the speed of blood collection and immediate centrifugation [49]. In the ten [13, 22, 24, 26, 29, 31–35] of 17 studies, blood was collected in sterile glass test tubes and immediately centrifuged at 3000 rpm for 10 min, while three [21, 28, 36] at 400 g for 12 min, one [27] at 2700 rpm for 12 min, one [30] at 3000 rpm for 12 to 14 min, one [37] in titanium tubes at 2800 rpm for 12 min, and one study [23] are unknown. In terms of usage, PRF was filled into the intrabony defects and used as a membrane to cover the defect in 15 studies, while only filled in the other two studies [13, 26]. (2) Great difference of teeth sites: six studies [23, 29–31, 34, 35] reported maxillary/mandibular single-rooted teeth or multirooted teeth, two [24, 33] reported maxillary/mandibular molar teeth, two [32, 36] only mandibular molar teeth, one [28] reported molar teeth without maxillary/mandibular types, one [37] only single-rooted teeth, one [27] reported maxillary/mandibular anterior teeth or premolars or molars, and four [13, 21, 22, 26] not mentioned. Most of the studies did not contain teeth with furcation involvement, but Bodhare et al. [24] reported intrabony defects with furcation involvement and three studies [13, 26, 32] not mentioned. (3) Baseline comparison between groups: there should be no difference in the baseline between groups, but seven studies [22, 24, 28, 31, 34, 35, 37] did not compare baseline differences between groups, although they have listed baseline data. (4) Blinding of participants: six studies [13, 22, 24, 27, 28, 36] did not state if participants were blinded, and these results might be affected duo to the Hawthorne effect.

RETRACTED

In the comparison of OFD+PRF and OFD alone, although the heterogeneity was high, forest plot of IBD depth reduction and BF% revealed that the studies are located on the right side of the vertical line, which indicated that all studies have affirmed the additional benefits of PRF, but the size of the benefits was not completely accurate because of the high heterogeneity. Therefore, there was ample evidence that OFD+PRF is superior to OFD alone. On the other hand, in the comparison of BG+PRF and BG alone, PRF also showed benefits in primary outcomes, but the benefit was smaller than that of PRF in the use of OFD. Although there was no heterogeneity, the evidence is not completely reliable due to the small number of studies.

The ease of preparation and cost-effectiveness of PRF offers a huge advantage, but the mechanical properties of PRF are poor. A study [50] to evaluate the mechanical properties of PRF found that PRF obviously lacked rigidity and degraded quickly, and the degradation rate after one week was about 36% of the initial mass. Because the epithelial barrier is needed to guide periodontal regeneration for at least 4 to 6 weeks [51], and the bone defects need longer maintenance time, so PRF cannot be used as a simple filling material or barrier membrane. PRF is more suitable to be used as an addition of periodontal regeneration surgery. At present, OFD is no longer regarded as periodontal regeneration surgery, and different combinations of strategies are gradually used for periodontal regeneration. Periodontal regeneration with many different regenerative materials, including barrier membranes, grafts, active biological compounds, and combinations of those, demonstrated significant clinical improvements in intrabony defects, far beyond those achieved with debridement only [4].

RETRACTED

In summary, based on the evidence and limitations in this review, it is suggested that more RCT studies are still required to explore whether PRF can enhance the regeneration effect of GTR or BG or combination of other modalities in the periodontal regenerative surgery. In the RCTs, it is recommended to carry out detailed design as follows to reduce bias as much as possible: adopt standardized PRF preparation process and surgical procedures, strictly recruit patients, use correct method of randomization and adequate allocation concealment, blinding of patients and outcome assessors, calibrate measurement results, and strengthen patient plaque control after operation.

## 5. Conclusion

In conclusion, current systematic review and meta-analysis has revealed that the use of PRF was significantly effective in the treatment of periodontal intrabony defects. The major findings suggest the following points:

1. In all the included studies, open flap debridement (OFD) combined with PRF was significantly better than OFD alone in intrabony defect depth reduction and bone fill % changes, but the size of the benefits was uncertain due to the high heterogeneity of the studies. In terms of PD reduction, CAL gain, and gingival margin level gain, the additional use of PRF seemed to be more effective compared to OFD alone
2. The combination of bone grafting (BG) and PRF will further increase the therapeutic effect of BG in intrabony defect depth reduction, PD reduction, CAL gain, and gingival margin level gain. The benefit of BG+PRF seemed to be less than OFD+PRF. But the small number of studies suggests a low degree of confidence and certainty in treatment effects
3. PRF seems to promote early wound healing in 1 week after periodontal surgery

## Figures and Tables

**Figure 1:** PRISMA flowchart for study selection.

**Figure 2:** Risk of bias summary of the included studies.

**Figure 3:** Forest plots for IBD depth reduction and BF% in the group OFD+PRF vs. OFD alone.

**Figure 4:** Forest plots for PD reduction, CAL gain, and GML gain in the group OFD+PRF vs. OFD alone.

**Figure 5:** Forest plots for IBD depth reduction, PD reduction, CAL gain, and GML gain in the group B +PRF vs. BG alone.

**Figure 6:** Funnel plot analysis of the studies. SE: standard error; MD: mean difference.

**Table 1:** General characteristics of the included studies.

Author (year)	Study design, blinded (duration)	Population			Intervention (number of surgical sites)	
		No. of participant baseline (end)	Age (mean/range)	Gender	Control	Test
Agarwal et al. (2016) [21]	Split-mouth, double blinded (12 months)	32 (30)	52 ± 7 (?)	14F/18M	OFD+DFDBA+saline (30)	OFD+DFDBA+PRF (30)
Ajwani et al. (2015) [22]	Split-mouth, single blinded (9 months)	20 (20)	30.5 (?)	10F/10M	OFD (20)	OFD+PRF (20)
Bajaj et al. (2017) [23]	Split-mouth, double blinded (9 months)	19 (17)	29.7 (20-30)	9F/10M	OFD (27)	OFD+PRF (27)
Bodhare et al. (2019) [24]	Split-mouth, single blinded (6 months)	20 (20)	35.9 (27-45)	9F/11M	OFD+bioactive glass (20)	OFD+bioactive glass+PRF (20)
Gamal et al. (2016) [25]	Split-mouth, single blinded (9 months)	30 (29)	39.6 ± 3.9 (28-51)	9F/21M	OFD+xenograft (9)	T1: OFD+xenograft+PRF (10); T2: OFD+xenograft+PRGF (10)
Kanoriya et al. (2016) [29]	Parallel, triple blinded (9 months)	108 (90)	39 (30-50)	55F/53M	OFD (30)	T1: OFD+PRF (30); T2: OFD+PRF+1% ALN (30)
Martande et al. (2016) [30]	Parallel, double blinded (9 months)	96 (90)	37.6 (?)	48F/48M	OFD (30)	T1: OFD+PRF (30); T2: OFD+PRF+1.2% ATV (30)
Patel et al. (2017) [26]	Split-mouth, double blinded (12 months)	13 (13)	44 ± 9 (?)	9F/4M	OFD (13)	OFD+PRF (13)
Pradeep et al. (2012) [34]	Parallel, double blinded (9 months)	54 (50)	36.8 (?)	27F/27M	OFD (30)	T1: OFD+PRF (30); T2: OFD+PRP (30)
Pradeep et al. (2015) [33]	Parallel, triple blinded (9 months)	126 (120)	41 (30-50)	60F/60M	OFD (30)	T1: PRF (30); T2: 1% MF (30); T3: OFD+PRF+1% MF (30)
Pradeep et al. (2016) [32]	Parallel, triple blinded (9 months)	90 (90)	35 (25-45)	45F/45M	OFD (30)	T1: OFD+PRF (30); T2: OFD+PRF+1.2% RSV (30)
Pradeep et al. (2017) [31]	Parallel, double blinded (9 months)	62 (57)	39.7 (?)	28F/34M	OFD (29)	T1: OFD+PRF (29); T2: OFD+PRF+HA (32)
Rosamma et al. (2012) [13]	Split-mouth, single blinded (12 months)	15 (15)	29.47 ± 7.65 (17-44)	9F/6M	OFD (15)	OFD+PRF (15)
Sezgin et al. (2017) [27]	Split-mouth, single blinded (6 months)	21 (15)	? (38-61)	7F/8M	OFD+ABBM (15)	ABBM+PRF (15)
Sharma et al. (2011) [35]	Parallel, double blinded (9 months)	42 (35)	35.34 ± 6.45 (30-50)	18F/24M	OFD (28)	OFD+PRF (28)
Thorat et al. (2011) [36]	Parallel, single blinded (9 months)	40 (32)	31.12 ± 2.06 (25-45)	18F/22M	OFD (16)	OFD+PRF (16)
Thorat et al. (2017) [28]	Split-mouth, single blinded (12 months)	18 (15)	25 ± 1.5 (?)	10F/8M	OFD (15)	OFD+PRF (15)
Ustaoğlu et al. (2020) [37]	Parallel, double blinded (9 months)	45 (45)	40 ± 8.37 (26-59)	22F/23M	OFD (15)	T1: OFD+PRF (15); T2: OFD+GTR (15)

OFD: open flap debridement; PRF: platelet-rich fibrin; DFDBA: demineralized freeze-dried bone allograft; PRGF: platelets rich in growth factors; ALN: alendronate; ATV: atorvastatin; PRP: platelet-rich plasma; MF: metformin; RSV: rosuvastatin; HA: hydroxyapatite; ABBM: anorganic bovine bone mineral; GTR: guided tissue regeneration.
